This article has been retracted.

# Cyber Risk Recommendation System for Digital Education Management Platforms

**DOI:** 10.1155/2022/8548534

**Published:** 2022-04-28

**Authors:** Xiufang Yin, Yanfang Chen

**Affiliations:** Zhengzhou Preschool Education College, Zhengzhou 450000, China

## Abstract

Covid-19 pandemic has ushered in a new school and academic year for students in a distance learning regime. This new daily routine was unprecedented and undoubtedly unusual, especially for the younger ones. At this point and at these ages, the risk of cyber fraud is even greater. The transition from the physical environment to the Internet took place quickly without the appropriate time to control potential risks and the proper information and training of teachers and students. Some common threats that need to be addressed to protect learners and their data when using e-learning methods are malicious remote access, malware, phishing, cyber fraud, etc. Considering the above situation, this work presents an innovative cyber risk recommendation system for digital education management platforms. The system in question is a distributed two-stage algorithm based on game theory and machine learning, which is trained by the constant change in the choice of recommendations by users to maximize security. We examine the algorithm's ability to simulate a user system in which everyone independently selects a user recommendation, assesses the environment and the implications of this choice, and then concludes whether it will continue to have that recommendation fixed. The methodology with which we have represented the digital e-learning system has been done with an approach that directly corresponds with their general view as a cyber-physical-social system. We consider the digital school as an environment that brings limitations, leading us to a pretty demanding personalization problem. Users coexist in this environment, in which everyone acts voluntarily but influences and is influenced by the surrounding environment. Our results lead us to conclude that this algorithm responds in a fully effective, flexible, and efficient way to the needs of protection and risk assessment of e-learning education systems.

## 1. Introduction

As the pandemic continues and educational institutions follow a hybrid education model (both physical and remote), the academic realm continues to attract the attention of digital criminals [1, 2]. The number of users who encountered threats disguised as popular online training/video conferencing platforms increased for all digital platforms. About 98% of the threats belonged to the not-a-virus category, divided into riskware and adware [3]. Adware bombards users with unwanted ads, while riskware consists of various files—from browser toolbars and download managers to remote management tools—that can perform multiple actions on the remote computer without the user's consent. Although much less than 1%, other types of more dangerous digital threats such as Trojans and Ransomware have also been reported [3]. Generally, users meet threats from unofficial websites that resemble the original platforms or spam emails and phishing campaigns presented as special offers or notifications by the platform or even by the e-learning institutions themselves [4, 5].

Under these conditions, the educational organizations that are directly affected try to organize, coordinate, and finally manage their organization's risk [6, 7]. Risk Management is defined as how organizations approach the risks associated with their activities and objectives to ensure timely and smooth development. The general idea is that the effort to achieve the goals of an organization is now intertwined with the effort to “repel” the various risks that threaten to hinder this endeavor, wherein, in this case, they concern the targeting of their educational mechanisms. Lack of confidence is eliminated, but it is constantly increasing due to the complexity of the digital world. Risk management allows organizations to prepare for this uncertainty, minimizing the risk they face before dealing with it. The ability to capture and control risks results in organizations making their decisions with greater certainty and confidence [8].

Digital risk analysis is a complicated and dynamic subject that requires a high level of skill in quantitative approaches, techniques, and instruments. It is an issue when risk management is implemented using out-of-date methods, especially in today's digital world. Cyber risk recommendation for digital education management platforms is proposed in this research, considering the above. We are dealing with a distributed two-stage method based on game theory and machine learning that continuously adapts to new proposals from users to maximize the safety of each one [6]. Replicating a user system in which each person makes their own choice, examines the consequences, and then makes their own choice again is what we are interested in. As a cyber-physical-social system, we consistently described the digital e-learning system with their overall vision [9]. We see the digital classroom as a constraining setting that forces us to confront a problematic personalization dilemma. Users cohabit in this ecosystem, where everyone acts on their own will but is influenced by their surroundings. Our findings concluded that our algorithm meets the protection and risk assessment demands of e-learning education systems as completely effective, adaptable, and efficient [10].

## 2. Related Literature

The danger of financial loss, interruption, or harm to an organization's reputation because of a breakdown of its information technology systems is known as cyber risk [8, 11]. A deliberate and unauthorized security breach to acquire access to information systems for espionage, extortion, or humiliation might be an example of such a danger. Also, unintended or unintentional security breaches may or may not represent an expose that has to be handled [12].

Amin [6] offered a pathway for evaluating cyber risk by creating a framework for a Bayesian network to simulate financial loss as a function of significant risk and resilience variables. Instead of taking a compliance approach to risk management, he took a valuation strategy. He employed a qualitative scorecard evaluation to analyze the extent of cyber risk exposure and the success of the organization's resilience strategies. He emphasized the uniqueness of risks and questioned the usual usage of actuarial models, which are typically used to analyze financial risk. There is a vast body of experience data.

The goal of Lassoued et al. [4] was to uncover the barriers to attaining quality in remote learning during the Coronavirus pandemic and to look into the many methods in which students continued their studies at home throughout the pandemic. They employed an exploratory, descriptive technique using a questionnaire given to both professors' and students' responses. According to the findings, teachers and students encountered self-imposed and educational, technological, budgetary, and organizational barriers. Universities blended traditional and new techniques of distance learning, as well as radio and television classes. After providing electronic publications via university websites, other institutions utilized the Internet to give lessons through different educational platforms or social networking sites to explain the lessons. When faced with similar or unanticipated obstacles in the future, the following recommendations were made to help in the study area and other areas to improve their ability to deliver high-quality distance learning.

Hakak et al. [2] looked at the harmful cyber activities linked to COVID-19 and various mitigating strategies. They also recommended an attack taxonomy to aid with risk management and mitigation in the future. They looked at COVID-19-themed hacks and divided them into four groups: service disruption, financial gain, stealing of information, and a piece of malware that took advantage of the pandemic fear, with subcategories inside each (e.g., malware, ransomware, phishing). They presented proposed mitigation methods using these categories. The cyberattack taxonomy and possible mitigation measures may also help design future pandemic cyberattack prevention efforts. They plan to expand on the suggested taxonomy and develop a risk management strategy for significant future crises.

Paris et al. [13] focused their research on the privacy problems that arose because of the pandemic's spread in higher education. They observed higher institutions' deployment of popular online learning platforms using critical informatics methodologies and theories to find numerous trends that emerged as a consequence of their implementation. They concluded their study by recommending measures to effectively manage the risks posed by higher education's usage of digital platforms, particularly those connected to privacy.

Thanou et al. [9] used quality of experience (QoE) to solve the challenge of integrating and analyzing the influence of visitor behavioral elements. User happiness has been frequently expressed using QoE, measured using correctly specified utility functions. The visitor quality of experience, as measured by a prospect-theoretic utility function, is greatly influenced by the total amount of time consumed in displays by all visitors, making their actions and choices interconnected and functioning more like a socially competitive environment. A game among visitors was designed and solved in a distributed method to identify the optimum time stay in exhibitions. The evaluation findings were provided in detail, emphasizing the functioning and superiority of the suggested framework while also giving obliging insights into visitor choices and behaviors under actual settings.

Based on the literature reviewed above, we can conclude that there is an open field for effective research in managing cyber risk in digital education management education platforms during pandemic crises, particularly in the manner presented in this study.

## 3. Proposed Approach

Given the uncertainty of documenting such a complex system, the proposed algorithmic approach focuses on modeling recommendations for users of educational applications, QoE, digital risk assessment, and the implementation of recommendations [14] in the user's system for their further protection [15]. More specifically, we deliberate an educational platform, where the best way to manage is to study, capture, and estimate the digital risk based on the time of each user's visit. We assume that users can choose between *R* different recommendations within the proposed platform.

For the present study, we will consider three different recommendations *R* = {*R*_*A*_, *R*_*B*_, *R*_*C*_}, while, in general, a digital program for managing educational activities may have more. Each of these recommendations offers users a different QoE and, at the same time, involves an extra degree of user engagement, which we will analyze in detail. We also denote the set of users as *N* = {1,…, *i*,…, *N*} of which each has its type of visit, namely ant, butterfly, fish, and grasshopper. The sets of users per type are denoted as *N*_*a*_, *N*_*b*_, *N*_*f*_, *N*_*g*_, and therefore, the group of users is *N*=*N*_*a*_ ∪ *N*_*b*_ ∪ *N*_*f*_ ∪ *N*_*g*_. Each of the classes has different behavior in terms of visit time, and how tolerant–careful–informed is the user in digital security about other users of the platform [16].

The time of each user's visit to the platform is symbolized as *t*_*i*_, and due to the characteristics of the platform (e.g., use of HTTPS) but also the personal characteristics and preferences–knowledge of each user, it is the upper and lower block, that is, *t*_*i*_^min^ < *t*_*i*_ < *t*_*i*_^max^. We also denote as *t*_−*i*_ the times of all other users coexisting simultaneously on the platform with user *i*, *i* ∈ *N*. Each different composition *R*_*x*_, *x* = *A*, *B*, *C*, and *R*_*x*_ ∈ *R* offers a different QoE to the user who chooses it. We call these QoE *Q*_*x*_, *x* = *A*, *B*, and *C* provided by the *R*_*A*_, *R*_*B*_, and *R*_*C*_ recommendations. Without compromising the generality, we assume that the values of these QoEs are sorted in a truly ascending order, that is, *Q*_*A*_ < *Q*_*B*_ < *Q*_*C*_, which indicates that the higher the recommendation identifier (*A*, *B*, *C*), the better the recommendation. A simple and effective metric that allows QoE verification for each user is the relative visit time ratio, which we define as [17, 18]

(1) $$\begin{array}{c} rt_{i}=\frac{t_{i}}{\sum \underset{j\neq i}{j\in N}t_{j}}, \end{array}$$

where the denominator is the total time that other users devote to their visit simultaneously as *i*. So we can easily observe that when the sum of the times of other users increases, then either the risk becomes higher, or the same number of users spend total time on the visit, which gives us an indication of the risk of misuse of the platform. In such a case, the user's *i* QoE deteriorates, either because there is a vast number of users on the platform, which means, for example, many shared files, augmented shared hyperlinks, or because some security issues are sidelined, resulting in increased inherent risk, for example, many interconnected external devices, access from unsafe media [19, 20].

We also assume that recommendations with increased QoE will lead users to the necessary time of the visit and the most basic security standards required since their stay will be more guided, and they will be offered a large amount of information in a short time, and in a more structured way. It is, therefore, natural for many users to ask for the most attractive recommendation, which will lead to a long wait for this recommendation due to the increased demand. Thus, the recommendations can be characterized by an additional congestion control parameter *c*_*x*_, *x* = *A*, *B*, *C*, representing the possible standby time for each proposal. This way, users should consider having a better recommendation, which may increase their QoE, but depending on how many have made the same choice, it can lead to a cost of waiting. The balance between the two should direct users to compromise and, therefore, to choose another recommendation. For our study, we undertake three different offers, which are the following [21–23]:

1. Recommendation *A* (*R*_*A*_): The platform has uploaded cyber security instructions. Users can follow these instructions in a short time without waiting for recommendations. However, they must comply with the platform's security rules without guidance and compliance checks. Thus, their perceived QoE (*Q*_*A*_) is limited as their security level for their browsing will be limited and possibly with significant security vulnerabilities.
2. Recommendation *B* (*R*_*B*_): A virtual guide is to assist users on the platform and provide explanatory and helpful information on critical security issues to look out for. Users form groups as they enter the platform, and the guide makes group recommendations at specific intervals. Therefore, users should suppose more time before starting their education platform to coordinate the team and carry out a group implementation process of the recommendations. However, their perceived QoE (*Q*_*B*_) will increase because they will have more structured information on critical security issues that concern them relatively quickly.
3. Recommendation *C* (*R*_*C*_): In addition to the features of the previous *R*_*B*_ recommendation, in *R*_*C*_, the guide provides users with information to implement–controlled by the user group. Depending on the number of teams that will be created and the different security levels that will have to be met, the completion times of the process will vary. Therefore, users will have to wait in even longer queues. However, the perceived QoE increases as the users digest the information even more.

According to the above description of the recommendations, we observe that the arrangement of QoE for each one is genuinely increasing, that is, *Q*_*A*_ < *Q*_*B*_ < *Q*_*C*_. In addition, more recommendations can be considered than the three we have proposed, following the same pattern, without compromising the generality. In addition, for the sake of equality and to support the concept of accessibility for more users on the platforms under consideration, we assume that all the above recommendations have the exact computational cost for users [20, 24]. Finally, the negatives for each recommendation can be summarized quantitatively in the computational cost of the congestion control parameter *c*_*x*_, *x* = *A*, *B*, *C* that we entered so that we will have *c*_*A*_ < *c*_*B*_ < *c*_*C*_.

The concept of a QoE function was adopted to represent the perceived satisfaction of each user as a function: the time devoted to the implementation of appropriate security measures, the recommendation chosen, and the satisfaction of their QoE prerequisites. A combined QoE function is adopted by each user and consists of the pure QoE component and the congestion control function. Pure QoE is expressed as the ratio of the QoE value achieved to the time spent using the platform. Thus, pure QoE increases if the user has achieved excellent QoE without devoting much time to using the platform. Note that the visit time is preferably for each user and is minimum and maximum blocked *t*_*i*_^min^ < *t*_*i*_ < *t*_*i*_^max^, as already mentioned. We also note that the optimal visit time will not always be *t*_*i*_^min^. Still, because QoE depends on the final recommendation choice and congestion on the platform (expressed by the total visit time of all users), QoE may be limited [25, 26].

Thus, the platform user expresses his flexibility regarding visit time (through the *t*_*i*_^min^ < *t*_*i*_ < *t*_*i*_^max^limits) and considers his perceived QoE to determine the optimal visit time. More specifically, the ideal QoE function is signified as an accounting function with a variable relative to the *rt*_*i*_ visit time, that is,

(2) $$\begin{array}{c} Q_{x}\cdot f_{i}^{y}\left(rt_{i}\right),\\ x=A,B,C,\\ y=a,b,f,g, \end{array}$$

where *y* denotes the four user categories *a*(nt), *b*(utterfly), *f*(ish), *g*(rasshopper). The function *f*_*i*_^*y*^(*rt*_*i*_), which we will refer to as the visiting efficiency function (VEF), represents user satisfaction and depends on the congestion on the platform at that time as well as how much time the user spends. Congestion is expressed solely by the time other users spend on the platform $\left(\sum_{\underset{j\neq i}{j\in N}}t_{j}\right)$. For the form of VEF, we chose the following sigmoid function [23, 24]:

(3) $$\begin{array}{c} f_{i}^{y}\left(rt_{i}\right)={\left(1-e^{-A_{y}rt_{i}}\right)}^{M_{y}}, \end{array}$$

where *A*_*y*_, *M*_*y*_, *y* = *a*, *b*, *f*, *g* are positive parameters that control the function's slope. Each of the four user types is characterized by a central relative visit time *rt*_*i*_, target, *y*, *y*=*a*, *b*, *f*, *g* which differs from species to species and is the turning point of the logistic function. The placement of the functions in the above order respects the characteristics of the visit types. We suppose that

(4) $$\begin{array}{c} rt_{i}^{\text{target},b}<rt_{i}^{\text{target},a}<rt_{i}^{\text{target},f}<rt_{i}^{\text{target},g}. \end{array}$$

The *butterfly*-type user can redirect his route to the platform in case of congestion as opposed to the type of *ant* that needs to check all possible checkpoints, and therefore,

(5) $$\begin{array}{c} rt_{i}^{\text{target},b}<rt_{i}^{\text{target},a}. \end{array}$$

The *fish* type user is waiting for the control procedures of the other group users to complete, so the satisfaction is limited. In contrast, *ant* user patiently completes all control procedures without complaint. So, we have

(6) $$\begin{array}{c} rt_{i}^{\text{target},a}<rt_{i}^{\text{target},f}. \end{array}$$

The *grasshopper* user has specific and limited security issues to resolve during his visit to the platform, so if he is late, his QoE decreases dramatically.

In general, if a user has less QoE than *rt*_*i*_^target,*y*^, then perceived satisfaction decreases rapidly. If, on the other hand, a user has a higher QoE than this, then the perceived QoE increases more slowly because the satisfaction conditions are met. Gathering the above observations, the combined QoE function can be expressed as [20, 22, 27]

(7) $$\begin{array}{c} Q_{i}\left(t_{i},t_{-i}\right)=\frac{Q_{x}\cdot f_{i}^{y}\left(rt_{i}\right)}{t_{i}}-c_{x}N_{x}^{k}e^{t_{i}},\;i\in N,\;x=A,B,C,\\ y=a,b,f,g,\;N=N_{a}\cup N_{b}\cup N_{f}\cup N_{g}. \end{array}$$

*N*_*x*_^*k*^ symbolizes how many users have chosen recommendation *x* at the time of calculation and is the population congestion factor that expresses a spatial weight concept in the weight of each recommendation. It is a way that gives us more control to adjust the cost of each recommendation according to the number of people our algorithm pretends, without having to change the cost values *c*_*x*_ which are inherent in the recommendations and do not make sense to change depending on how large the total number of users examined.

The penetration of a composition *R*_*x*_, *x* = *A*, *B*, *C* is expressed as the ratio of the total combined QoE of the users. They have chosen the composition *R*_*x*_ to the total achieved combined QoE of all users present on the platform for the specific observation moment *τ*. We define the penetration of a recommendation as [28, 29]

(8) $$\begin{array}{c} p_{x}\left(\tau \right)=\frac{\sum_{\begin{array}{c} R_{x}\\ N \end{array}}^{N}Q_{x}\cdot f_{i}^{y}\left(rt_{i}\right)}{\sum_{\begin{array}{c} i=1\\ \forall R_{x}\in R \end{array}}^{N}Q_{x}\cdot f_{i}^{y}\left(rt_{i}\right)}. \end{array}$$

The above process allows the systematic approach of controlling and assessing the risks associated with the activities of users participating in e-learning platforms. The focus of efficient risk management is to identify and manage these risks to ensure a robust environment that can be causally assessed. The categorization and control of users in groups increase the probability of success of the educational organization's overall security and defense objectives. It should be noted that the proposed procedure can be visualized as a three-dimensional network of random walks.

A random walk is a random process in mathematics that depicts a path made up of an unpredictably large number of unexpected steps on a particular mathematical space random walk on a regular lattice is a prominent random walk model in which a probability distribution determines the position of each stage. A probability distribution determines the location of each step. If you take a simple random walk, the place can only jump to neighboring lattice sites, which results in a lattice path being formed. In an introductory symmetric random walk on a locally finite lattice, the probability of a location jumping to each of its immediate neighbors is the same as the likelihood of the place jumping to the location's close neighbors. A three-dimensional network of random walks is shown in Figure 1 [30, 31].

The properties of transience and reproducibility (true and not) in this three-dimensional network of random walks are class properties. If a state *x* has one of these properties, then all states of class *x* belong to have the same property. It is reasonable that short sequences are open (and vice versa; every open class is passing). In contrast, iterative classes are closed (the inverse is not valid–generally finite closed classes are iterative), which means that a Markov chain is created that allows them to appear in transient states with a probability of 1 and after a finite number of steps, to return to a repetitive state. Hence, they are essentially forever in the repetitive state class [32, 33].

Based on the above formulation, and assuming that the Markov chain is nondegradable, genuinely repetitive, and nonperiodic, then regardless of its initial distribution, we have [30, 32, 34]

(9) $$\begin{array}{c} P\left[\frac{V_{n}\left(i\right)}{n}⟶\pi \left(i\right),\forall i\in S\right]=1. \end{array}$$

So, if the transition from one situation to another situation entails a fee or some cost (negative fee) of the form,

(10) $$\begin{array}{c} R_{n}=R_{n}\left(X_{n-1},X_{n}\right),\;n\in \mathbb{N}. \end{array}$$

for the *n*-th step, then we have a total reward in the first *n* steps equal to

(11) $$\begin{array}{c} C\left(n\right)=\sum_{s=1}^{n}R_{s}\left(X_{s-1},X_{s}\right). \end{array}$$

While for the average reward in one step it applies

(12) $$\begin{array}{c} \underset{n⟶\infty }{\lim}\frac{C\left(n\right)}{n}=\sum_{j}r_{j}\cdot \pi_{j}. \end{array}$$

In conclusion, we can say that the risk assessment can reveal from the early stages of implementing a distance learning system the severe security gaps that the organization should address and the possible ways to avoid them. The developed risk management procedures described are ongoing throughout the educational project, with digital risk management applying to all individual projects, from the smallest (implemented by one person) to vast and complex. Many issues can be addressed in advance and allow the project manager to determine a specific course using the proposed cyber risk recommendation system for digital education management platforms [7].

## 4. Modeling

To model the proposed system, we implemented a specialized scenario to verify the location of the user's actions when using an e-learning platform. Before starting their browsing, users entering the platform select a recommendation to guide their browsing based on a machine learning framework. Users act as cellular automata who gain information and experience from their previous actions as the time of the algorithm progresses. At the end of the algorithm, they will have chosen the final recommendation, which will be the one that will guide them during their browsing on the platform.

These automata can listen to their environment while keeping a history of their past decisions to make beneficial decisions in the future that will lead them to optimize their QoE. The necessary information needed to decide on the recommendation they will make is the time of the visit and the values of the combined QoE of the previous iteration *τ* of the machine learning part of the algorithm. In addition to the above parameters, each user has advised the input of each recommendation *R*_*x*_, *x* = *A*, *B*, *C* of all users, that is, *p*_*x*_ (*τ*), to make the final decision and action *a* (*τ*). Given the actions of the users regarding the selection of the recommendation, the users take part in a distributed noncooperative game for the determination of the visit time, played in each repetition of the machine learning algorithm, to regulate the optimal visit time as well as the corresponding value of their QoE [33, 35, 36].

Therefore, the algorithm consists of these two repetitive decision parts, one for selecting the recommendation and one for choosing the visit time, and is done before the users visit the platform. In addition, we emphasize that the algorithm is executed every time a new user enters the platform, considering the history of all previous users who are already on the platform. The algorithm's execution time is relatively short, which is helpful since it is executed while users are waiting for the application to start.

The platform environment consists of *R*_*x*_, *x* = *A*, *B*, *C*, *R*_*x*_ in *R* different recommendations, and *N* users can be studied as a learning system, where users act as learning machines and respond to their environment to decide which recommendation to choose. Each user/automaton is learning *i*, *i* ∈ *𝒩*, *𝒩*=*𝒩*_*a*_ ∪ *𝒩*_*b*_ ∪ *𝒩*_*f*_ ∪ *𝒩*_*g*_ for each iteration *τ* of the machine learning system and has a set of actions *a*_*A*_, *a*_*B*_, *a*_*C*_. This set of actions represents the different choices that users can make regarding the recommendation. To adopt what action to take for each iteration *τ*, users consult the output *β* (*τ*) = *Q* (*τ*), *t* (*τ*) of their environment, where *Q* (*τ*) and *t* (*τ*) are vectors that contain the combined QoE and the visit time of each user for the snapshot *τ*. The output *β* (*τ*) = *Q* (*τ*), *t* (*τ*) is determined after the execution of the time management part.

Combining the selected actions of the users and the reaction of the system in the form of QoE, we calculate the probability of rewarding. This probability is the penetration of the *R*_*x*_ composition and is expressed by the relation [11, 37, 38]

(13) $$\begin{array}{c} p_{x}\left(\tau \right)=\frac{\sum_{i=1}^{N}Q_{x}\cdot f_{i}^{y}\left(rt_{i}\right)}{\sum_{\begin{array}{c} i=1\\ R_{x}\in R \end{array}}^{N}Q_{x}\cdot f_{i}^{y}\left(rt_{i}\right)}. \end{array}$$

The probability of each user's action is expressed as a vector which in turn describes the probability that user *i* selects the *R*_*x*_, *x* = *A*, *B*, *C* recommendation, and following the automata learning model, this probability is updated in each round as follows:

(14) $$\begin{array}{c} {\mathrm{Pr}}_{i,x}\left(\tau +1\right)={\mathrm{Pr}}_{i,x}\left(\tau \right)-b\cdot p_{x}\left(\tau \right)\cdot {\mathrm{Pr}}_{i,x}\left(\tau \right),\;x^{\left(\tau +1\right)}\neq x^{\left(\tau \right)},\\ {\mathrm{Pr}}_{i,x}\left(\tau +1\right)={\mathrm{Pr}}_{i,x}\left(\tau \right)+b\cdot p_{x}\left(\tau \right)\cdot \left(1-{\mathrm{Pr}}_{i,x}\left(\tau \right)\right),\;x^{\left(\tau +1\right)}=x^{\left(\tau \right)}, \end{array}$$

where *b*, 0 < *b* < 1 is a parameter that controls the convergence time of the process. The equation represents the probability that the user must choose in (*τ* + 1) a composition different from the one in (*τ*). At the same time, it also describes the probability that the user continues to prefer the same composition, that is, *x* (*τ* + 1) = *x* (*τ*). As for the loading of the selection probabilities of each recommendation, in the absence of any prior knowledge of the personal preference of each user, the algorithm initially considers all possibilities equally. Finally, we point out that each user converges on the recommendation that can offset the cost of waiting in line and the limitations in the visit times that everyone has.

Given the recommendation option, each user *i*, *i* ∈ *N*, aims to select the optimal visit time to maximize their QoE. Therefore, the above problem can be expressed as a distributed QoE maximization problem in terms of visit time as

(15) $$\begin{array}{c} \underset{t_{i}}{\max}Q_{i}\left(t_{i},t_{-i}\right),\\ \tau .\omega .t_{i}^{\text{Min}}<t_{i}<t_{i}^{\text{Max}},\\ \forall i\in N,x=A,B,C,\\ y=a,b,f,g,N=N_{a}\cup N_{b}\cup N_{f}\cup N_{g}. \end{array}$$

Due to the distributed nature of the optimization problem and the selfish nature of the users in terms of optimizing their QoE, a game theory approach is applied to determine the optimal time for each. We denote as *G*={*N*, *T*_*i*_, *Q*_*i*_} the noncooperative visit time selection game, where *N* is the set of players, that is, the users of the platform, *T*_*i*_=[*t*_*i*_^Min^, *t*_*i*_^Max^] is the strategy space of the *i*-th user and *Q*_*i*_ the corresponding QoE function of this user. To decide in detail on the solution, we will recall the concept of Nash equilibrium. To ensure the existence and uniqueness of the Nash equilibrium, we must show that the *Q*_*i*_ function of each user is a convex function for *t*_*i*_. A function *Q*_*i*_ can be strictly convex if for every pair of different *t*_*i*_ − *t*_*i*_′ belonging to the convex set *T*_*i*_, with 0 < *λ* < 1,

(16) $$\begin{array}{c} Q_{i}\left(t_{i}^{\prime }\right)>Q_{i}\left(t_{i}\right)⟹Q_{i}\left(\lambda \cdot t_{i}+\left(1-\lambda \right)\cdot t_{i}^{\prime }\right)>Q_{i}\left(t_{i}\right). \end{array}$$

The combined QoE function of user *i*, *i* ∈ *N*, *N*=*N*_*a*_ ∪ *N*_*b*_ ∪ *N*_*f*_ ∪ *N*_*g*_ is convex in the strategy interval Τ_*i*_′ corresponding to the interval of the relevant time ratio [19, 33, 36, 39].

(17) $$\begin{array}{c} rt_{i}\in \left(\frac{\ln\;M}{A},rt_{B}\right),\;rt_{B}\in \left(\frac{\ln\;M_{y}}{A_{y}},\frac{\ln\;10^{4}M_{y}}{A_{y}}\right). \end{array}$$

Consequently, the Nash equilibrium point of the game *G*={*N*, *T*_*i*_, *Q*_*i*_} exists and is unique in the corresponding strategy interval.

To prove the curvature of the combined QoE function of users, we will consider the sign of the second derivative for *t*_*i*_.

(18) $$\begin{array}{c} \frac{\partial^{2}Q_{i}}{\partial t_{i}^{2}}=g\left(rt_{i}\right)+h\left(rt_{i}\right)-c_{x}N_{x}e^{t_{i}}, \end{array}$$

where

(19) $$\begin{array}{c} g\left(rt_{i}\right)=\frac{2Q_{x}}{t_{i}^{3}}{\left(1-e^{A_{y}rt_{i}}\right)}^{-My}\left[-M_{y}A_{y}e^{-A_{y}rt_{i}}rt_{i}+1-e^{-A_{y}rt_{i}}\right]\times \alpha ,\\ h\left(rt_{i}\right)=\frac{M_{y}A_{y}^{2}Q_{i}}{t_{i}^{3}}{\left(1-e^{-A_{y}rt_{i}}\right)}^{-2M_{y}}e^{-A_{y}rt_{i}}rt_{i}^{2}\left(M_{y}e^{-A_{y}rt_{i}}-1\right). \end{array}$$

Since *g*(*rt*_*i*_) is continuous, we conclude that

(20) $$\begin{array}{c} g\left(rt_{i}\right)<0,\;\forall rt_{i}\in \left(\frac{\ln\;M_{y}}{A_{y}},rt_{B}\right). \end{array}$$

By default, the Nash equilibrium of the noncooperative game should satisfy the following:

(21) $$\begin{array}{c} t_{i}^{*}={\text{BR}}_{i}\left(t\right)=\arg\max Q_{i}\left(t_{i},t_{-i}\right). \end{array}$$

We, therefore, conclude that the overall convergence of the noncooperative time management game at the Nash equilibrium point, under the proposed best response function, is guaranteed.

## 5. Results

To evaluate the algorithm, we will study the importance of the various parameters for the system and their effect on the solutions provided by the algorithm. Precisely, we must first determine the input of the algorithm, which consists of the following:

1. The strategy field, *T*_*i*_=[*t*_*i*_^Min^, *t*_*i*_^Max^] represents the minimum and maximum time available to the student *i* ∈ *N*
2. Cost values *c*_*x*_, *x*=*A*, *B*, *C* of each recommendation
3. The values QoE *Q*_*x*_*x*=*A*, *B*, *C* of each composition
4. The total number of visitors *N*
5. The visit type of each visitor *y*_*i*_=*a*, *b*, *f*, *g*.
6. The force *k* of the population congestion parameter *N*_*x*_^*k*^
7. The four visit efficiency functions *f*.

By executing the algorithm, we obtain as a result for each visitor the *R*_*i*_ recommendation chosen by the visitor, the QoE value of each visitor, and the suggested visit time of each visitor. Therefore, to evaluate the correctness of the algorithm results, we will observe these three outputs for each scenario. In addition, we will assess the time performance of the algorithm depending on the increase in the number of visitors and the change of the merging parameter *b* in the machine learning model [40–42].

To evaluate the algorithm's results in assigning a recommendation to each visitor, we first studied a system with ten (*N*=100) visitors. The following two diagrams show the final QoE price for each visitor. Specifically, in Figure 2, the QoE value is depicted for each visitor and average QoE with the forced assignment of recommendations.

Figure 2 shows the result of the game if we omit the machine learning part and assign to all visitors the seemingly best recommendation *C*.  Figure 3 shows the QoE value for each visitor and average QoE from the use of the proposed algorithm, with the same parameters as in the above case.

We have marked a pair (*R*, *y*) above each value in both cases. *R* represents the final composition selected for visitor *i* while *y* is the visitor type [*a* (nt), *b* (utterfly), *f* (ish), *g* (rasshopper)]. All tests were made in the Google Colab environment using GPU: Nvidia K80/T4, GPU Memory 12 GB; GPU memory clock: 1.59 GHz; and performance: 4.1 TFLOPS.

Comparing the two charts above, we observe that the algorithm has avoided assigning the best recommendation to all users and has set the recommendations so that all visitors are satisfied as far as possible. We also observe that the algorithm leads to QoE values that avoid excessive satisfaction and excessive dissatisfaction, bringing visitor satisfaction levels close to the average value. In addition, both in Figure 3 and in all the results we got, the visitors—*ants* and the *butterflies*—are consistent among the most satisfied. This approves that these two types of visitors show the most patience, both in the queues and during their visit.

Finally, the effect of overcrowding can be seen in Figure 2, but if we look closely, it is also evident in Figure 3. More specifically, taking as an example visitors 4 and 5 in Figure 3, we observe that a “better” composition does not imply a better QoE. Visitors 4 and 5 are of the *fish* type, and while four has received recommendation *A* which is more straightforward than *B*, it nevertheless has a better QoE than 5. This is because for recommendation *A* the tail is only three visitors while for *B* it is four. Therefore, because *fish*-type visitors are impatient, 4 has less anticipation and thus more satisfaction.

We then considered a system with one hundred (*N*=100) visitors evenly distributed with the four types of visits (25 visitors per type).  Figure 4 shows the result of the average QoE value and visit time for each of the visit types.

The results are representative of the selection of visit efficiency functions. More specifically, *butterfly* and *ant* visitors have the highest QoE, while the most difficult to satisfy *fish* and *grasshopper* types have the lowest QoE. Visit times are also typical of the distribution given by the functions in question. This is because the breaking points of the functions are progressively more right for each type of visitor. This results in the best QoE value being at a higher time value. The above result reveals the exceptional importance of the functions in the configuration of the problem and the modeling of the types of visitors. In conclusion, visit efficiency functions are the basic configuration of the algorithm that encodes the behavior of the four types of visits.

Figure 5 offerings the total number of visitors who have selected each recommendation as to the timing *τ* of the machine learning part of the algorithm progresses.

As it turns out, the game in the early stages is more active as the machine learning loop pushes visitors to review their recommendation options frequently. Then, the changes are reduced, and the visitors come to their final recommendation with certainty. We also notice that the number of repetitions is relatively small, implying a short execution time. In addition, we observe that, in the time range between 50 and 70, the algorithm's response to the dominance of a recommendation can be seen where, for that snapshot, it pushes the revision of the recommendations to the next round of recurrence machine learning. It is worth noting that we considered that the visitor system does not receive additional visitors in the scenarios we examined. Therefore, the stabilization we observe is final. However, if the system received new visitors during the algorithm's execution, this stabilization would cease with the entry of unique visitors and would return much faster. This is because, as we have shown, the equilibrium point exists and is secured.

We, therefore, conclude that the presence of the machine learning loop is significant for the operation of the algorithm. Without visitors being seen as automata learning, there would be no feedback loop that allows the algorithm to know the system as a whole. The circle of machine learning is the one that enables the elimination of such nonuniform solutions. In particular, in the event of an internal situation, the value of the penetration factor *p*_*x*_ in the linear law of probability renewal will give recommendation *C* a minimal value. Consequently, in the next iteration of the problem of finding the optimal visit time, many visitors will have been pushed away from recommendation *C*. Thus, the algorithm has avoided this undesirable outcome.

## 6. Conclusions

This paper presented an innovative cyber risk recommendation system for digital education management platforms. The system implements and proposes a distributed two-step algorithm based on game theory and machine learning, which is trained by the continuous change in the choice of recommendations by users to maximize the provision of the desired level of digital security and the corresponding risk these platforms capture. The proposed algorithm is an innovative effort in distance learning education systems. It is a fully automated risk assessment system with which educational institutions can ensure the levels of digital security and the quality of the user experience in a thorough and adaptable way. The simplicity of implementation, as well as the low computational complexity, is what makes it extremely useful and functional. However, the low computational complexity hides in the background of the need for careful configuration, that is, there is a delicate balance between the fast implementation time and the time it needs to be configured. The variety of usage and configuration options allows the respective educational organizations to organize the right balance for the individual digital educational platform. This algorithm can be applied based on their individual needs and priorities.

Given the plethora of customization, many new paths can be drawn after studying the applications of the proposed system. The cost parameters, the benefit of the recommendations, and the congestion parameter should be directly linked to the platform and the individual quality and risk characteristics that characterize it to optimize the implementation of the algorithm and strengthen the potential of each organization to offer each recommendation. Finally, given the framework of machine learning and automata learning, convergence step *b* needs additional study in terms of its importance in terms of the behavior of machines (visitors) in conjunction with the implementation time, which we studied in this paper. More specifically, it is worth investigating whether a small refresh parameter attributes a feature to how visitors respond to the system of recommendations. In other words, a big step may mean a quick and imperfect way of updating the visitors' opinion, but, in some cases, depending on the way the cost of the recommendations is organized, it may be more desirable. In this way, additional knowledge can be obtained as to which price to choose and whether it will be in the high or low range.

This research's future directions are primarily concerned with the investigation and extension of the model with inherent capabilities of optimizations processing for the automated system to fully utilize the powers of more comprehensive dependencies of modeling learning systems with increased accuracy and efficiency. The potential examination of the impact of such a grouping methodology on risk assessment and management development, compared to standard ways of separation, is particularly intriguing, as is the possibility of doing such research utilizing nonparametric machine learning methods in the future.

## Figures and Tables

**Figure 1:** Random walks on multilayer networks.

**Figure 2:** QoE value for each visitor and average QoE (forced assignment of recommendations).

**Figure 3:** QoE value for each visitor and average QoE (forced by the proposed algorithm).

**Figure 4:** Average QoE and average visiting time vs. visiting time.

**Figure 5:** Visitors per recommendation for each timeslot *τ*.

## Data Availability

The data used in this study are available from the author upon request.
